# A Systematic Review of Weight-Based Metoprolol for Acute Atrial Fibrillation with Rapid Ventricular Rate

**DOI:** 10.1155/2023/3138064

**Published:** 2023-04-15

**Authors:** Alexandra Burum, Jasmine Carino, Mackenzie McBeth, Nephy Samuel, Trager D. Hintze

**Affiliations:** Department of Pharmacy Practice, Texas A&M Irma Lerma Rangel School of Pharmacy, 159 Reynolds Medical Bldg, MS 1114, College Station 77843-1114, TX, USA

## Abstract

Atrial fibrillation (AF) is the most common cardiac arrhythmia encountered in the emergency department (ED) and when patients present in acute AF with rapid ventricular rate (RVR), it can result in significant morbidity and mortality. Primary treatment modalities are aimed at rate control with the two most common agents being intravenous metoprolol and diltiazem. Some evidence suggests that diltiazem may be more effective at controlling rate in these patients; however, the dosing strategies, pharmacologic differences, and study designs may play a role in the observation of these differences. The purpose of this article is to review the evidence for using weight-based metoprolol in the treatment of AF with RVR. The vast majority of studies comparing metoprolol and diltiazem for the treatment of acute AF with RVR compare a flat dose of metoprolol to a weight-based dose of diltiazem. Following a comprehensive review, only two studies have compared a weight-based dosing strategy of intravenous (IV) metoprolol versus IV diltiazem for this disease state. Overall, the two studies only contained 94 patients and failed to meet power. Beyond differing dosing strategies, differences in pharmacokinetics between the two medications (like the onset of action and metabolism) could have played a role in the differences observed in the studies. Further studies are warranted to provide better guidance on which agent should be used in the treatment of acute AF with RVR.

## 1. Introduction

Atrial fibrillation (AF) is a type of cardiac arrhythmia that occurs when abnormal electrical activity causes the atria to contract irregularly and out of sync with the ventricles. AF results in nearly half a million hospitalizations and contributes to more than 158,000 deaths per year. It is also the most common type of arrhythmia seen in the emergency department. [1] It is estimated that in 2030 the incidence and prevalence of AF will increase to 2.6 million and 12.1 million cases, respectively, primarily due to the aging population in the United States. [2] Roughly 60–70% of all AF cases seen in the emergency department present with rapid ventricular response (RVR) which can lead to significant morbidity and mortality. In AF with RVR, the abnormal activity of the atria causes the ventricles to contract too rapidly. This results in increased myocardial oxygen demand and reduced cardiac output as the ventricles are unable to fill completely. Patients with AF with RVR can experience tachycardia, angina, dyspnea, dizziness, or syncope. Complications of untreated AF with RVR can include hemodynamic instability, tachycardia-induced cardiomyopathy, heart failure, arterial thromboembolism, cerebrovascular accidents, and death [3].

In the emergency department, the primary treatment strategy is to reduce the heart rate (i.e., rate control). In AF with RVR, rate control is important as it reduces morbidity and decreases the potential for developing tachycardia-induced cardiomyopathy. According to the 2014 AHA/ACC/HRS Atrial Fibrillation Guidelines, intravenous administration of a beta blocker such as metoprolol or a nondihydropyridine calcium channel blocker such as diltiazem is recommended to slow ventricular heart rate in the acute setting. Yet, currently there is no guidance for selecting one agent over the other [3]. Beta blockers provide rate control by blocking sympathetic tone, and historically, were the most commonly selected agents. Many clinicians opt for diltiazem as there is some evidence to suggest it may be more effective [4, 5]. However, the dosing strategies (weight-based vs flat dosing), pharmacologic differences, and study designs may play a role in the observation of these differences [6]. The purpose of this article is to review the evidence for using weight-based metoprolol in the treatment of AF with RVR.

## 2. Methods

A comprehensive electronic search was conducted to uncover all peer-reviewed articles related to the topic of weight-based metoprolol for the treatment of acute AF with RVR. The literature review was conducted based on the principles from the 2020 Preferred Reporting Items for Systematic Reviews and Meta-Analyses guidelines [7]. PubMed and Ovid databases were systematically searched using the phrases: “Intravenous metoprolol for atrial fibrillation with rapid ventricular rate” and “Weight-based intravenous metoprolol for atrial fibrillation with rapid ventricular rate.” In addition, the reference sections from the sourced articles were screened to identify other publications. Articles that met inclusion criteria for the review were original prospective trials, published in the English language, utilized a weight-based dosing strategy of medications for the treatment of acute AF with RVR, and compared intravenous metoprolol to diltiazem. Titles and abstracts from the initial literature searches were screened for relevance and eligibility. The full-text review was then completed by two authors independently. Data extracted by the authors included, as available: doses of metoprolol and diltiazem, dosing strategies of the medications, rates of efficacy, rates of hypotension and bradycardia, and patient demographics related to weight. Statistically significant *p* values, if reported in the article, are included in the results section.

## 3. Results

Review of the literature yielded 3 studies comparing weight-based intravenous (IV) metoprolol versus IV diltiazem in atrial fibrillation with rapid ventricular rate. One study was not published in English and not retrievable, thus it was omitted.

The first trial that studied weight-based metoprolol dosing in the acute treatment of AF with RVR was a prospective double-blind study published in 2005 by Demircan and colleagues. Patients either received IV diltiazem 0.25 mg/kg (maximum dose 25 mg) or IV metoprolol 0.15 mg/kg (maximum dose of 10 mg). This trial included 40 patients with 20 patients per treatment arm. The primary outcome was time to successful treatment which is defined as an HR of <100bpm, a decrease in HR by 20% (minimum of 120bpm), or conversion to normal sinus rhythm. This trial also included a secondary outcome of a decrease in blood pressure. The mean percentage decrease in HR was significantly higher in the diltiazem group at 2, 5, 10, 15, and 20 minutes. The number of people who reached treatment success at 2 minutes was 50% in diltiazem and 15% in the metoprolol group (*p* < 0.05). There was no statistical difference in the amount of people who reached treatment success at 5, 10, 15, and 20 minutes. There was no statistical difference in the decrease of blood pressure between the two interventions and while both drugs caused a decrease in blood pressure, none of the patients had hypotension (SBP <90 mmHg) [8].

The second study was published more recently in 2015 by Fromm and colleagues. Their prospective double-blind trial compared IV diltiazem versus IV metoprolol in the management of AF with RVR. This study had a total of 54 patients: 25 patients receiving 0.25 mg/kg of diltiazem (maximum dose 30 mg) and 29 patients assigned to 0.15 mg/kg of metoprolol (maximum dose of 10 mg). The primary outcome was HR < 100 bpm within 30 minutes of drug administration. Secondary outcomes were HR < 60 bpm and SBP <90 mmHg. In the first 5 minutes, 50% of the diltiazem group and 10.7% of the metoprolol group reached the target heart rate (*p* < 0.005). At 30 mins, 95.7% of the diltiazem group and 46.4% of the metoprolol group achieved the goal heart rate (*p* < 0.001). There was no difference between the treatment groups in terms of hypotension (*p* = 0.199) or bradycardia (*p* = 0.462) [9].

## 4. Discussion

The articles reviewed comparing intravenous diltiazem and metoprolol for the acute treatment of AF with RVR suggest diltiazem may be more effective than metoprolol at achieving rate control targets. Two meta-analyses, by Lan and colleagues in 2021 and by Sharda and colleagues in 2022, suggest similar outcomes. However, only 3 out of 17 studies in the Lan meta-analysis and 2 out of 14 in the Sharda meta-analysis, totaling only 11% and 5% of the studied population, respectively, compared weight-based metoprolol and diltiazem [4]. The remaining studies compare flat dose metoprolol versus weight-based diltiazem, so it is important to question whether diltiazem only appears more efficacious due to the difference in dosing strategies.

The 2014 AHA/ACC/HRS Atrial Fibrillation Guidelines recommend the administration of a flat dose of metoprolol 2.5–5 mg IV bolus given over two minutes or a weight-based dose of diltiazem 0.25 mg/kg IV bolus given over two minutes for the treatment of AF with RVR in the acute setting. [3] While a flat dose for metoprolol is what is recommended, patients may benefit from receiving a weight-based dosing regimen instead. The administration of a flat dose of metoprolol could be resulting in the underdosing of patients. For example, a 5 mg dose of metoprolol in a 70 kg patient is 0.07 mg/kg. A 5 mg dose of metoprolol in a heavier 120 kg patient is 0.04 mg/kg. The recommended weight-based dose for metoprolol, however, is 0.15 mg/kg, so in both cases the patient would be underdosed. Using a weight-based dose for both medications may be more useful in determining the agent best suited for rate control of AF with RVR.

At present, there is insufficient data comparing weight-based metoprolol and diltiazem for the treatment of AF with RVR. Only the two studies, by Demircan and Fromm, compare metoprolol 0.15 mg/kg to diltiazem 0.25 mg/kg and caution should be exercised when interpreting results, as both studies have limitations. Both studies have a small patient population size with a combined total of 94 participants, of which, only 49 received the weight-based metoprolol dosing. The study by Fromm and colleagues failed to meet power. The statistical analysis needed 200 participants to meet 80% power, but the study only enrolled a total of 54 patients. It is unclear if the study by Demircan and colleagues met power. Furthermore, the article by Demircan and colleagues only collected data up to 20 minutes after administration and so stopping the monitoring at this time may not have shown the full effects of metoprolol as this agent has a delayed onset of action [8, 9].

The limitations of these studies may not be the only thing affecting the results. It is important to take into consideration the pharmacokinetic differences between the two medications. Metoprolol has an onset of action of approximately 20 minutes after IV administration while diltiazem has an onset of action of approximately 3 minutes after administration [10, 11]. This difference in onset of action could explain why both studies found that diltiazem reached primary endpoints quicker, but failed to show differences at the later time points [8, 9]. In terms of metabolism, diltiazem is both a substrate and an inhibitor of CYP3A4 and thus can result in some drug-drug interactions [11]. Further metoprolol is metabolized by CYP2D6 which is subject to genotype variability resulting in poor and ultra-rapid metabolizers [10, 12, 13]. Incidence of ultra-rapid metabolizers has an incidence of up to 29% in the African American population which can affect the efficacy of the medication, while in the Asian population up to 12% are poor metabolizers which can lead to more adverse reactions [13].

It is difficult to determine how clinicians are choosing whether to treat with metoprolol or diltiazem in practice. The two biggest side effects of both the drugs are bradycardia and hypotension, however, neither meta-analysis by Lan (2021) or Sharda (2022) show a statistical difference in the incidence of these adverse events [4, 5]. Some of the other side effects to consider for diltiazem are edema, hyperglycemia, and severe skin reactions whereas metoprolol can cause exercise intolerance, bronchospasms, and mask symptoms of hypoglycemia. According to a retrospective cohort study conducted by Hines and colleagues, the only predictors of the selection of metoprolol instead of diltiazem were a history of AF, diabetes mellitus, and the patient having been prescribed a beta blocker prior to ED presentation [6]. Patients prescribed a calcium channel blocker prior to ED presentation which were a negative predictor of the selection of beta blocker as initial therapy. Comorbidities such as a history of heart failure, volume overload, a positive troponin test, and chest pain were not predictors of the selection of metoprolol over diltiazem. Likewise, a history of asthma or COPD did not result in the selection of diltiazem over metoprolol.

While the articles reviewed seem to suggest diltiazem as the preferred agent in the treatment of AF with RVR, using weight-based metoprolol dosing over the current flat dosing strategy may increase the efficacy of metoprolol [4, 5, 8, 9]. It is important to note, however, that metoprolol may still not be preferred in the acute setting due to the delayed onset of about 20 minutes compared to diltiazem's onset of 3 minutes. Furthermore, since metoprolol is primarily metabolized by CYP2D6, it may not be the agent of choice for patients that are poor metabolizers or ultra-rapid metabolizers. On the other hand, in cases in which CYP3A4 inhibitors are to be avoided, metoprolol would be the agent of choice. Since there is the possibility of increased efficacy when using weight-based metoprolol dosing compared to flat dosing more research is needed to compare the two dosing strategies, especially in populations with extreme body weights such as patients with obesity as there may be a benefit of an increased dose for these larger patients.

## 5. Conclusion

Some of the published literature on the acute treatment of AF with RVR suggests diltiazem may be the preferred agent, though it is important to recognize the overall paucity of the literature and limitations of the published studies. Some pharmacokinetic parameters may favor diltiazem for AF with RVR but using weight-based metoprolol over the current flat dosing strategy may prove beneficial, especially in extremes of body weight. Considering the limitations of the studies that compare weight-based metoprolol versus diltiazem, more research would provide better guidance on which agent should be used in the treatment of atrial fibrillation with rapid ventricular rate.
